RETRACTED

# Impact of Small Incision Reduction and Suture Linked with Functional Appliance of Sufferers with Irrecoverable TMJ Anterior Disc Displacement

**DOI:** 10.1155/2022/7196599

**Published:** 2022-09-26

**Authors:** Xiaotong Wei, Wei Yan, Anjun Sun, Hao Wang, Wei Wang

**Affiliations:** Oral and Maxillofacial Surgery Department, Cangzhou Central Hospital, Hebei Province, Cangzhou City 061000, China

## Abstract

**Methods:**

90 patients with irreducible ADD of TMJ treated from August 2020 to August 2021 were acquired in our hospital. They were randomly divided into control group and trial group randomly. There were 45 patients in each group. The sufferers in the control group were treated with oral drug therapy and small incision reduction and suture, while those in the trial group were treated with small incision reduction and suture linked with functional appliance. The pain score, dysfunction, joint function recovery, facial improvement, and clinical impacts of the two groups were contrasted.

**Results:**

Compared with that in the control group at 1 week, 4 weeks, and 6 months after therapy, the pain score in the trial group was markedly higher. After therapy, in the two groups, maximum vertical opening (MVO), left lateral excursion (LLE), and right lateral excursion (RLE) levels were markedly higher than those in the control group. The MRI score of the trial group was markedly higher than that of the control group at 1 week, 4 weeks, and 6 months after therapy, and the total effective rate of the trial group was markedly higher than that of the control group.

**Conclusion:**

The use of small incision reduction and suture linked with functional appliance in the therapy of sufferers with irreducible ADD of TMJ is beneficial to relieve pain, promote the recovery of body function, and contribute to the recovery of joint function.

## 1. Introduction

Anterior disc displacement (ADD) of temporomandibular joint (TMJ) is a common disease, and its pathogenesis is complicated, which is markedly related to environmental, genetic, and acquired genetic factors [1, 2]. ADD of TMJ refers to the obstruction of TMJ of the brain, which leads to the disorder of internal structure and the disorder of internal structure of TMJ, which seriously affects the life of sufferers [3, 4]. The occurrence of the disease is relatively sudden. With the continuous evolution of the ADD of the TMJ, there will be abnormal mouth opening, resulting in the obstruction of joint function, the damage of the joint strangulation, and the local pain in the joint area, which will seriously affect the quality of life of the sufferers [5, 6]. At present, clinical medical research has found that the irreducible ADD of the TMJ will cause local pain in the articular disc and maxillofacial region, which will seriously affect the patient's living ability, cause joint deformation and serious drop in joint height, and then lead to facial deformity, which will have a great impact on the patient. It occurs frequently in young people [7]. Conservative therapy for sufferers, the course of the disease cure cycle is long, and for those with severe symptoms, it will affect the appearance of sufferers [8, 9]. Therefore, we should find a more scientific and accurate therapy, so as to effectively improve the satisfaction of sufferers. Small incision reduction and suture can effectively reduce the pain of sufferers, thus effectively reduce the difficulty of operation, thus improve the clinical impact, promote the growth and repair of joints, and improve the healthy life and ability of sufferers. The recovery of neurological function plays a very important role [10–12]. This study formulated the relevant therapy methods for the ADD of the TMJ and could explore the therapy methods of the sufferers with ADD of the TMJ. In this study, 90 sufferers with ADD of the TMJ admitted in our hospital from September 2019 to December 2021 were selected as the trial group, which were reported as follows.

RETRACTED

## 2. Materials and Methods

### 2.1. General Information

90 patients with irreducible ADD of the TMJ treated from August 2020 to August 2021 were acquired in our hospital. They were randomly divided into control group and trial group. There were 45 patients in each group. Among them, there were 20 males and 25 females in the trial group, the age was 35-60 years old, the average age was (46.36 ± 8.31) years, the height was 161-183 cm, the average height was (165.79 ± 5.78 cm), the weight 61 kg-81 kg, the average weight (67.61 ± 6.21) kg, and the body mass index 21-30 kg/m^2^, the average body mass index (25.63 ± 2.23) kg/m^2^. There were 23 males and 22 females in the control group, the age was 38-62 years old, the average height was (45.46 ± 10.01) years, the height was 162-182 cm, the average height was (164.46 ± 3.98 cm), the weight 63 kg-84 kg, the average weight was (66.46 ± 6.82) kg, and the body mass index was 21-34 kg/m^2^, the average was (26.69 ± 2.35) kg/m^2^. There was no noteworthy divergence in sex, age, and other general data (*P* > 0.05), which was comparable.

### 2.2. Inclusion and Exclusion Criteria

Inclusion criteria: the pain of TMJ lasted for more than 3 months; the pain site was mainly located in sufferers with ADD of the TMJ, which can be radiated above the joint; the main manifestation of pain was joint pain; the ADD of the TMJ could not be reduced; the medical records such as past history and medication history were complete; informed consent was signed. Exclusion criteria: ADD of the TMJ caused by various visceral diseases; ADD of the TMJ caused by deformity, tumor, fracture, or other trauma; pregnant and lactating women; long-term bedridden sufferers; disturbance of consciousness; complicated with dysfunction of the heart, kidney, lung, and other important organs.

RETRACTED

### 2.3. Research Methods

The sufferers in the control group received routine therapy for ADD of the TMJ; they were treated with modified small incision surgery, and the subcutaneous tissue was cut into the subtemporal anterior membrane, cut the front of the vein, so as to cut the superficial layer of infratemporal membrane, resection along the vein. So as to protect the inferior middle temporal vein and the temporal branch of the nerve, injected normal saline into the articular cavity, so as to effectively protect the middle artery, exposed the joint capsule, added physiological saline into the supraarticular cavity, opened the attachment point of the joint disc from the inside, released the front part, reset the joint part, separated along the internal tendons, and reset the joint disc, so as to effectively improve the reduction function of the joint disc, put the suture out at the inside and outside, after it was introduced into the forearm of the external auditory canal, after threading the suture, the sutured part was sutured at the joint, and finally put the drainage tube into it, sewed the part tightly, and removed the suture after operation, so as to effectively improve the postoperative reexamination position of the sufferer and observe the recovery of the scar.

The sufferers in the trial group were treated with small incision reduction and suture linked with functional appliances. The sufferers were in the prone position, with a thin pillow on their abdomen, and its abdomen was covered with a thin pillow. Aligned the sufferer's jaw, performed the blade at the front, performed the operation at the midline, and used its forward extension reduction for correction, adjusted the activity every day, adjusted the grinding tool with the corrector, and the adjustment height was 1 mm. Configured it 24 hours a day. Adjusted the mold from front to back, and the mold adjustment height was 1 mm until the mold pressing part was effectively adjusted, the posterior teeth were adjusted with the help of the tube sleeve device, and the anterior jaw was effectively adjusted, removed the corresponding cannula and adjusted the jaw, the orthodontic apparatus was removed. Physical therapy was conducted, once a day, and lasted for 10 days.

RETRACTED

### 2.4. Trial Indicators

(I) Pain score: visual analogue score (VAS) [13] was used to evaluate the pain degree of the two groups before therapy, 1 week, 4 weeks, and 6 months after therapy. The higher the score, the more severe the pain. (II) Mandibular movement: the standard of mandibular movement [10] was used to evaluate the painless maximum vertical opening (MVO), left lateral excursion (LLE), and right lateral excursion (RLE) before and after therapy. (III) Clinical curative impact evaluation: Excellent: after therapy, the low back pain disappeared, the movement was unimpeded, and the sufferers were able to work and live normally; Good: the pain almost disappeared, the activity was slightly limited, but had little impact on work and life; Fair: the symptoms were improved to a certain extent, but the pain existed, affecting work and life; Poor: the symptoms were not improved or even aggravated. Total efficiency rate = (Cases of good + Cases of fair)/Total cases. (IV) MRI index observation: before therapy, 1 week, 4 weeks, and 6 months after therapy, the sufferers in the two groups were observed with MRI, so as to effectively evaluate the position of their joint disc, and different therapy methods were used for sufferers with joint disc in different positions, so as to determine their MRI index and evaluate the postoperative repositioning

### 2.5. Statistical Processing

The data of this study were analyzed by SPSS22.0 statistical software. The trial indexes selected in the study were expressed by mean ± standard deviation ($\bar{x}\pm s$). Independent sample *t*-test was used for inter-group comparison, and paired sample *t*-test was used for intra-group comparison. *P* < 0.05 meant the difference was statistically significant.

## 3. Results

### 3.1. Contrasted the VAS Scores of the Two Groups

There was noteworthy divergence in the VAS score and the change trend of VAS score among the trial group and the control group (*P* < 0.05). Before therapy, there was no noteworthy divergence in VAS pain score between the two groups (*P* > 0.05). The VAS pain score of the trial group was markedly higher than that of the control group at 1 week, 4 weeks, and 6 months after therapy (*P* > 0.05), as shown in Table 1.

### 3.2. Comparison of Mandibular Conditions between the Two Groups

Before therapy, there was no noteworthy divergence in the levels of MVO, LLE, and RLE between the two groups (*P* > 0.05), but the levels of MVO, LLE, and RLE in the two groups strengthened markedly after therapy (*P* < 0.05), and the levels of MVO, LLE, and RLE in the trial group were markedly higher than those in the control group (*P* < 0.05), as shown in Table 2.

### 3.3. Clinical Efficacy

The total effective rate of sufferers in the trial group was 91.11%, which was markedly higher than that in the control group (*P* < 0.05), as shown in Table 3.

RETRACTED

### 3.4. MRI Score

Before therapy, there was no noteworthy divergence in MRI score between the two groups (*P* > 0.05). The MRI score of the trial group was markedly higher than that of the control group 1 week, 4 weeks, and 6 months after therapy (*P* < 0.05), as shown in Table 4.

## 4. Discussion

As a common clinical disease, the etiology of ADD of the TMJ is complicated, and some sufferers have clear pathological causes and imaging manifestations, such as difficulty in mouth opening, serious abnormality in mouth opening, and pain in the joint area. However, the vast majority of patients have joint pain during the onset, which seriously affects the quality of life of patients [14, 15]. In the clinic, ADD of the TMJ arthropathic pain is more common. The sufferer's articular disc can be restored due to long-term abnormal stress or other minor injuries. The failure of reduction of the articular disc will cause facial pain and dysfunction and cause serious damage to the articular disc. In addition, its facial deformities seriously affect the quality of life of the patients. At present, the therapy of ADD of the TMJ is often lack of pertinence, and the curative impact is poor, which brings serious problems to sufferers and their families [16–18]. At present, the clinical therapy of ADD of the TMJ is mainly small incision reduction and suture, which will bring some disadvantages and cannot be treated accurately. With the gradual development of medical technology, the improvement of small incision reduction and suture in the past therapy process, which can effectively treat the changes in the lower position of sufferers, has now made a major breakthrough and achieved noteworthy therapeutic impacts [19–22]. In the process of therapy with functional instruments, both its accuracy and feasibility can be well guaranteed, which provides a sufficient scientific basis for guiding the therapy of sufferers' mandibular joints, and can effectively solve sufferers' pain feelings [23].

In this study, the VAS pain score of the trial group was markedly higher than that of the control group at 1 week, 4 weeks, and 6 months after therapy; it showed that using small incision reduction and suture linked with functional appliance to treat sufferers with irreducible ADD of the TMJ could reduce the degree of pain and duration of pain, played a good role in promoting the prognosis of sufferers, and improved the quality of life of sufferers [24–26]. It was consistent with the study of small incision reduction and suture in the treatment of ADD of the TMJ, relieving pain and improving joint function by Xing et al. [27]. From the clinical efficacy of the two groups of sufferers, the total effective rate of the trial group was 91.11%, markedly higher than that of the control group, indicating that the therapy impact of small incision reduction and suture linked with functional appliance on sufferers with irreducible ADD of the TMJ was better, and the total effective rate of cure was higher. From the MRI scores of the two groups of sufferers, the MRI scores of sufferers with chronic low back pain in the trial group were markedly higher than those in the control group 1 week, 4 weeks, and 6 months after therapy. This was consistent with the higher effective rate of joint reduction compared with the reduction and suture of TMJ under small incision by He et al. confirmed [28]. These conclusions indicated that the therapy of sufferers with irreducible ADD of the TMJ with small incision reduction and suture linked with functional appliances could promote the recovery of sufferers' physical functions, reduce the recurrence of sufferers' conditions, and control the prognosis better.

RETRACTED

To sum up, the therapy of sufferers with irreducible ADD of the TMJ with small incision reduction and suture linked with functional appliance is conducive to reducing the degree of pain, improving the pain situation of sufferers, avoiding some postoperative complications, promoting the recovery of normal functions, and improving the quality of life of sufferers (Figure 1).

## Figures and Tables

**Figure 1:** Abstract diagram.

**Table 1:** VAS pain score ($\bar{x}\pm s$, score).

Grouping	Instances	Before therapy	One week after therapy	4 weeks after therapy	6 months after therapy
Trial group	45	4.39 ± 1.17	1.07 ± 0.43^∗^	0.81 ± 0.32^∗^	0.50 ± 0.12^∗^
Control group	45	4.54 ± 1.11	1.40 ± 0.52^∗^	1.12 ± 0.47^∗^	0.72 ± 0.26^∗^
*t* value		0.624	3.281	3.657	5.154
*P* value		0.534	0.002	0.0004	<0.0001

Note: Contrasted with before therapy, ^∗^*P* < 0.05.

**Table 2:** Mandibular condition of two groups of sufferers ($\bar{x}\pm s$, mm).

Grouping	MVO (mm)		LLE (mm)		RLE (mm)	
	Before therapy	After therapy	Before therapy	After therapy	Before therapy	After therapy
Trial group (*n* =45)	22.86 ± 5.28	43.46 ± 7.15^∗^	7.59 ± 0.52	8.36 ± 0.42^∗^	6.85 ± 1.12	7.78 ± 0.53^∗^
Control group (*n* =45)	22.90 ± 5.54	28.61 ± 7.17^∗^	7.56 ± 0.43	7.89 ± 0.34^∗^	6.74 ± 1.29	7.08 ± 0.76^∗^
*t* value	0.351	9.872	0.298	5.835	0.432	5.608
*P* value	0.972	0.001	0.766	<0.0001	0.667	<0.0001

Note: Contrasted with before therapy, ^∗^*P* < 0.05.

**Table 3:** Clinical efficacy [*n* (%)].

Grouping	*n*	Excellent	Good	Fair	Poor	Total efficiency rate
Trial group	45	23 (51.11)	18 (40.00)	3 (6.67)	1 (2.22)	41 (91.11)
Control group	45	15 (33.33)	17 (37.78)	10 (22.22)	3 (6.67)	32 (71.11)
*x* ^2^ value						5.874
*P* value						0.015

RETRACTED

**Table 4:** MRI scores ($\bar{x}\pm s$, score).

Grouping	Instances	Before therapy	One week after therapy	4 weeks after therapy	6 months after therapy
Trial group	45	36.45 ± 7.32	27.30 ± 7.65^∗^	26.51 ± 6.85^∗^	27.31 ± 7.56^∗^
Control group	45	37.10 ± 6.81	21.43 ± 7.78^∗^	19.73 ± 5.46^∗^	21.33 ± 7.20^∗^
*t* value		0.436	3.609	5.192	3.842
*P* value		0.664	<0.0001	<0.0001	<0.0001

Note: Contrasted with before therapy, ^∗^*P* < 0.05.

## Data Availability

The datasets used and analyzed during the current study are available from the corresponding author upon reasonable request.
